# A novel *EIF4ENIF1* mutation associated with a diminished ovarian reserve and premature ovarian insufficiency identified by whole-exome sequencing

**DOI:** 10.1186/s13048-019-0595-0

**Published:** 2019-12-06

**Authors:** Minying Zhao, Fan Feng, Chunfang Chu, Wentao Yue, Lin Li

**Affiliations:** 1 Department of Reproductive Medicine, The First Hospital of Shijiazhuang, 36 Fanxi Road, Shijiazhuang, 050011 Hebei China; 2 Department of Basic Medical Sciences, School of Medicine, Tsinghua University, Haidian, Beijing, 100084 China; 3 Department of Gynecology, Beijing Obstetrics and Gynecology Hospital, Capital Medical University, Chaoyang, Beijing, 100026 China; 4 Central Laboratory, Beijing Obstetrics and Gynecology Hospital, Capital Medical University, Chaoyang, Beijing, 100026 China

**Keywords:** Diminished ovarian reserve, Whole-exome sequencing, EIF4ENIF1, Premature ovarian failure

## Abstract

**Background:**

To dissect the genetic causes underlying diminished ovarian reserve (DOR) and premature ovarian insufficiency (POI) within a family.

**Methods:**

Whole-exome sequencing of the proband was performed and DOR and Sanger sequencing was carried out to validate presence of the variant in the proband and her mother. In silico algorithms were used to analyze the mutational effect of the variant. PSIPRED (PSI-blast based secondary structure PREDiction) was used for predicting mutated protein secondary structures.

**Results:**

Using whole-exome sequencing, we found that the proband carries the mutation c.2525A > C;p.Q842P in *EIF4ENIF*, a POI-related gene. Through Sanger sequencing, we found that the proband’s mother also carries the same mutation. Online bioinformatics analysis suggests that the mutation is a pathogenic mutation. Secondary structural biology prediction analysis indicates that the mutation either causes the destruction of the α-helical structure around the mutation site or reduces the α-helix.

**Conclusions:**

This mutation is the second novel mutation of *EIF4ENIF1* that has been identified in POI patients. This study thus provides a theoretical basis for POI genetics and POI clinical genetic counseling.

## Background

Ovarian development consists of a series of elaborate developmental processes, including primordial germ cell migration and development, meiosis, and folliculogenesis. The ovarian reserve is related to the number and quality of the remaining oocytes. As such, diminished ovarian reserve (DOR) is used to describe women of reproductive age with regular menstruation cycles whose response to ovarian stimulation or reproductive capacity is less than that of women of comparable age. DOR can be identified based on an abnormal ovarian reserve test (antral follicular count < 5–7 follicles or anti-Mullerian hormone < 0.5–1.1 ng/mL) [1]. DOR is different from premature ovarian insufficiency (POI), which is characterized by at least 4 months of amenorrhea or oligomenorrhea, elevated follicle-stimulating hormone (FSH) levels (> 25 IU/L), and low estradiol. The prevalence of POI is ~ 1% in the general population [2]. Several factors, including chromosomal abnormalities, Fragile X premutations, point mutations, autoimmune disorders, and medical or surgical interventions, contribute to the onset of POI. However, the causes of POI for most women remain unclear, although unexplored genetic factors may partially explain some POI cases. POI and DOR share a common pathogenesis and are both related to abnormal ovarian reserves. We thus hypothesize that DOR may represent an early stage and partial manifestation of POI.

From a genetic point of view, POI is a heterogeneous disease [3]. The pathogenic molecular mechanism of POI has been thought involve mutations in genes involved in several developmental processes, including primordial germ cell survival [4], DNA repair and meiotic recombination [5–12], oocyte transcription and translational control during folliculogenesis [13–20], granulosa cell development [21–25], and oocyte mitochondrial function [26, 27].

*EIF4ENIF1*, or eukaryotic translation initiation factor 4E nuclear import factor 1, is a nucleocytoplasmic shuttle protein that is enriched in P-bodies for transport of the translation initiation factor eIF4E. In addition, EIF4ENIF1 can competitively prevent the productive binding of eIF4E to eIF4G, thereby reducing protein synthesis by regulating ribosomal delays through interfering with the interaction between eIF4E and eIF4G [28]. EIF4ENIF1 can thus control access of the 5′ cap of specific mRNAs by ribosomes and mediate translational repression [29, 30]. Previous studies have shown that EIF4ENIF1 is a part of a large CPEB (Cytoplasmic Polyadenylation Element Binding) translation inhibitor RNP (RiboNucleoProtein) complex in *Xenopus laevis* oocytes [31]. In mouse oocytes, EIF4ENIF1 is essential for breakdown of the nuclear envelope and the resumption of meiosis [32]. Moreover, in a large French-Canadian family [20], seven women affected with POI possessed a heterozygous premature stop codon (Ser429*) in *EIF4ENIF1* that was not present in the unaffected members, suggesting a dominant mode of inheritance of POI-causing *EIF4ENIF1* mutations [20]. *EIF4ENIF1* is therefore a good candidate gene for investigation to determine its role in POI and ovarian reserve abnormalities.

In this study, we recruited a family in which the proband was diagnosed with DOR and whose mother was a POI patient. We then used whole-exome sequencing to dissect the genetic causes underlying DOR in this family.

## Methods

### Patients

All procedures involving human participants were performed in accordance with the ethical standards of the Ethics Committee of the First Hospital of Shijiazhuang and the 1964 Helsinki declaration and its later amendments. Written informed consent was obtained from each participant. The proband (Fig. 1a, II-1) with DOR was recruited from the First Hospital of Shijiazhuang. The proband developed DOR in 2018 at the age of 28. The hormone levels of the proband were as follows: follicle-stimulating hormone, 8.71 IU/L; luteinizing hormone, 2.93 IU/L; estradiol, 62 pmol/L; testosterone, 0.48 nmol/L; prolactin, 8.32 ng/mL; and anti-Mullerian hormone, 1.67 ng/mL. Ultrasound imaging of the left (Fig. 1b) and right (Fig. 1c) ovaries showed no antral follicles and one antral follicle, respectively. In addition, the proband’s mother (Fig. 1a, I-2) developed amenorrhea at the age of 39.

**Fig. 1:** The proband and her pedigree. **a** The proband with DOR and her mother with POI. The black arrow indicates the proband. **b** Ultrasound imaging of the proband’s left ovary lacking antral follicles. **c** Ultrasound imaging of the proband’s right ovary containing only one antral follicle

### Whole-exome sequencing and data analysis

Genomic DNA was extracted from peripheral blood using a QIAamp DNA Mini Kit (Qiagen, Valencia, CA, USA). Whole-exome sequencing (WES) was performed as previously described [33]. A two-step process was used for filtering variants. First, rare and novel variants (minor allele frequency < 1%) were selected. Minor allele frequencies were analyzed based on data in the Exome Aggregation Consortium (ExAC, http://exac.broadinstitute.org/), 1000 Genomes (http://browser.1000genomes.org/index.html), Genome Aggregation Database (gnomAD, http://gnomad.broadinstitute.org/), and ESP6500 (http://evs.gs.washington.edu/EVS/) databases. Second, only frameshift, nonsense, missense, and splicing-site variants were retained.

### Sanger sequencing validation

WES results were validated using Sanger sequencing. For the *EIF4ENIF1* (c.2525A > C:p.Q842P) variant, forward (5′-ATGAAGCAAACGATGGTTCC-3′) and reverse (5′-TAGGGGATTGACTGGATTGG-3′) primers were used for PCR amplification and Sanger sequencing. DNA products were evaluated using electrophoresis with an ABI 3730 XL DNA sequencer (Applied Biosystems, Bedford, MA).

### Protein secondary structure predictions

PSIPRED [34] was used to predict protein secondary structures. PSIPRED generates secondary structure predictions using up to four feed-forward neural networks and PSI-BLAST outputs, which are then used to find related sequences and build a position-specific scoring matrix. The generation of a sequence profile is performed by PSI-BLAST then normalized by PSIPRED. The prediction of an initial secondary structure is done by a neural network, while a second neural network is used to filter the structure predicted by the first network. PSIPRED then predicts the secondary structure with the highest score.

## Results

### WES analysis of the proband and sanger sequencing validation

The proband was diagnosed with DOR, while her mother was diagnosed with POI, suggesting that genetic factors may play an important role in observed ovarian disfunction. WES was performed to analyze the potential genetic causes of proband DOR. WES data was filtered to retain frameshift, splice-site, missense, and nonsense variants while excluding variants with allele frequencies > 1% in the whole-exome or whole-genome databases (ExAC, gnomAD, ESP6500, and 1000 Genomes). This led to identification of the variant c.2525A > C;p.Q842P in the POI-related gene *EIF4ENIF1*, which had previously been associated with POI in a study analyzing a large pedigree [20]. The proband variant c.2525A > C was confirmed using Sanger sequencing (Fig. 2a) and appears to have been inherited from her mother, not her father (Fig. 2a).

**Fig. 2:** Analysis of the *EIF4ENIF1* variant. **a** Sanger sequencing validation of the heterozygous c.2525A > C mutation in the *EIF4ENIF1* gene. The red arrow indicates the mutation site. **b** Amino acid sequence alignment of EIF4ENIF1 from different species. The red arrow indicates the mutated amino acid. Glutamine at position 842 is 100% conserved in all species

### In silico analysis of the *EIF4ENIF1* variant

By performing sequence alignment analysis, we found that Q842 is highly conserved across species ranging from humans to zebrafish (Fig. 2b), suggesting that Q842 plays an important role in EIF4ENIF1 protein function. The allele frequency of c.2525A > C is 0.0000084, 0.00001634, 0, and, 0 in the ExAC, gnomAD, ESP6500 and 1000 Genomes databases, respectively (Table 1). This suggests that the c.2525A > C variant is very rarely found in the general population. Five of six online prediction tools for mutation effects suggest that Q842P is a disease-causing mutation (Table 1). Moreover, analysis using the Constraint Metrics Z score for missense variation suggests that *EIF4ENIF1* gene is intolerant to variation, with z = 1.95 and pLI = 1.00 (http://exac.broadinstitute.org/gene/ENSG00000184708). This indicates that the *EIF4ENIF1* gene has fewer variants than expected and that the heterozygous variant found in *EIF4ENIF1* may be pathogenic. Therefore, in summary, all in silico analyses performed predicts that the c.2525A > C;p.Q842P variant may be a pathogenic mutation associated with DOR and POI.

**Table 1:** In silico analysis of *EIF4ENIF1* mutation

Variants	Amino acid change	Polyphen-2^a^	SIFT^b^	PROVEAN^c^	Mutation Taster^d^	SNPs&GO^e^	FATHMM-MKL^f^	gnomAD^g^	ExAC^h^	1000 Genomes^i^	ESP6500^j^
c.2525A > C	p. Q842P	Probably damaging (0.996)	Damaging (0.002)	Deleterious (− 3.21)	Disease causing (0.999)	Neutral (0.247)	Damaging (0.983)	0.00001634	0.0000084	0	0

^a^Polyphen-2. Prediction Scores range from 0 to 1 with high scores indicating probably or possibly damaging

^b^SIFT, i.e., Sorting Intolerant From Tolerant. Scores vary between 0 and 1. Variants with scores close or equal to 0 are predicted to be damaging

^c^PROVEAN. Variants with scores lower than − 2.5 (cutoff) are predicted to be deleterious

^d^Mutation Taster. The probability value is the probability of the prediction, i.e., a value close to 1 indicates a high ‘security’ of the prediction

^e^SNPs&GO. Probability: Disease probability (if > 0.5 mutation is predicted Disease)

^f^FATHMM-MKL. Values above 0.5 are predicted to be deleterious, while those below 0.5 are predicted to be neutral or benign

^g^Frequency of variation in total of gnomAD database

^h^Frequency of variation in total of ExAC database

^i^Frequency of variation in 1000 Genomes database

^j^Frequency of variation in ESP6500 database

### Modeling of the secondary structure of EIF4ENIF1 Q842P

The structure of a protein is extremely important for its biological function. We therefore predicted the secondary structure of EIF4ENIF1 (721-900aa) using PSIPRED 4.0.1 (Fig. 3a) and found that the Q842 site was crucial for α-helix formation (red cylinder). Q842 is located at the beginning of the helix and sequence conservation analysis showed that Q842 is conserved across species. These results thus illustrate the importance of Q in the formation of EIF4ENIF1 secondary structure and function. In the variant detected in our study, Q was mutated to P. By using computer-based calculations, we identified two possible results of this mutation (Fig. 3b). This mutation may result in the conversion of the α-helix in the wild type protein to a random coil or may change the length of the α-helix. P is thus considered problematic for helix formation, especially when present in the middle of the sequence. Due to the molecular structure of proline, the Q842P mutation changes the structural stability of the α-helix. Such structural changes can then affect protein-protein interactions or signal transduction, leading to misregulation of normal gene transcription.

**Fig. 3:** Structural analysis of the variant. **a** Secondary structure prediction of EIF4ENIF1 by PSIPRED 4.0.1. The straight line represents a coil and the cylinder represents an α-helix. The star indicates the Q842. **b** Modeling of the secondary structure of EIF4ENIF1 Q842P. The upper image shows how Q842P could change the α-helix into a coil while the lower image shows how Q842P may change the length or form of the α-helix

## Discussion

In this study, we identified an *EIF4ENIF1* heterozygous variant in a patient with DOR using WES. Moreover, we found that this patient inherited the variant from her mother, who suffers from POI. Bioinformatics analysis suggests that the variant c.2525A > C;p.Q842P may be a pathogenic allele. Additionally, secondary structure modeling suggests that Q842P may change the original α-helix structure.

The *EIF4ENIF1* mutation found in this study is a heterozygous mutation, in line with its dominant inheritance. The genetic mode of inheritance of POI in this study is consistent with that described in the previously published literature [20]. Two possible mechanisms can be used to explain the presence of this mutation: haploinsufficiency or the dominant-negative effect. However, previously published studies [20] indicate that the haploinsufficiency mechanism is more likely since these studies found a premature stop codon (p.Ser429*) in a variant of *EIF4ENIF1* while our study identified a point mutation (p.Q842P) in *EIF4ENIF1*. Since we have not done the relevant functional experiments, we cannot determine whether the effect of this point mutation completely eliminates protein function. However, the haploinsufficiency mechanism is more likely the cause of the effects of heterozygous *EIF4ENIF1* mutations since the EIF4ENIF1 protein has not been reported to function as a dimer. In general, when a protein can function as a dimer, the mutation found in that protein will have a dominant negative effect. EIF4ENIF1 inhibits protein translation by binding to EIF4E [35], decreases in levels of EIF4ENIF1 lead to partial decreases in EIF4E inhibition, which may result in increased protein translation and enhanced mRNA stability.

## Conclusions

In conclusion, our study identified a rare mutation of the *EIF4ENIF1* gene in a family exhibiting DOR and POI. Online bioinformatics analysis suggests that this mutation is a pathogenic mutation. Moreover, secondary structural biology prediction analysis suggests that this mutation either causes the destruction of the α-helical structure around the mutation site or a reduction in α-helix length. This mutation is the second novel mutation of *EIF4ENIF1,* identified in POI patients. This study therefore provides new information on POI genetics and a novel gene locus for use in genetic counseling for POI and related diseases.

## Data Availability

The datasets used and/or analyzed during the current study are available from the corresponding author upon reasonable request.
